The article "Motion of Lumbar Endplate in Degenerative Lumbar Scoliosis Patients with Different Cobb Angle In Vivo: Reflecting the Biomechanics of the Lumbar Disc" was published in 2022. Journal: Biomed Res Int.

# Motion of Lumbar Endplate in Degenerative Lumbar Scoliosis Patients with Different Cobb Angle In Vivo: Reflecting the Biomechanics of the Lumbar Disc

**DOI:** 10.1155/2022/8745683

**Published:** 2022-10-14

**Authors:** Fei Xu, Shuai Jiang, Longjie Wang, Xiangyu Hou, Siyu Zhou, Zhuofu Li, Zhuoran Sun, Da Zou, Weishi Li

**Affiliations:** ^1^Orthopaedic Department, Peking University Third Hospital, No. 49 North Garden Road, Haidian District, Beijing 100191, China; ^2^Peking University Health Science Center, No. 38 Xueyuan Road, Haidian District, Beijing 100191, China; ^3^Beijing Key Laboratory of Spinal Disease Reasearch, China; ^4^Engineering Research Center of Bone and Joint Precision Medicine, Ministry of Education, Beijing, China

## Abstract

**Objective:**

To evaluate the influence of degenerative lumbar scoliosis (DLS) with different Cobb angles and degenerative discs on the range of motion (ROM) of the lumbar endplates during functional weight-bearing activities in vivo. *Summary of Background*. DLS data might influence spinal stability and range of motion of the spine. Altered lumbar segment motion is thought to be related to disc degeneration. However, to date, no data have been reported on the motion patterns of the lumbar endplates in patients with DLS in vivo.

**Methods:**

We recorded 42 DLS patients with the apical disc at L2-L3 and L3-L4. Patients were divided into A group with a coronal Cobb angle >20° (number: 13; 62.00 ± 8.57 years old) and group B with a coronal Cobb angle <20° (number: 28; 65.79 ± 6.66 years old). Patients' discs were divided into a degenerated disc group (III-V) and a nondegenerated disc group (I-II) according to the Pfirrmann classification. Computed tomography (CT) was performed on every subject to build 3-dimensional (3D) models of the lumbar vertebrae (L1–S1), and then the vertebras were matched according to the dual fluoroscopic imaging system. The kinematics of the endplate was compared between the different Cobb angle groups and the healthy group reported in a previous study and between the degenerative disc group and nondegenerative disc group by multiway analysis of variance.

**Results:**

Coupled translation at L5-S1 was higher than other levels during the three movements. During the flexion-extension of the trunk, around the anteroposterior axis, rotation in group A was higher than that in the control group at L2-L3 and L3-L4 (6.62 ± 3.61 mm vs 4.36 ± 2.55 mm, 5.01 ± 3.19 mm; *P* < 0.05, *P* < 0.05). During the left-right bending of the trunk, around the mediolateral axis, rotations in groups A and B were higher than those in the control group at L5-S1 (17.52 ± 11.43°, 17.25 ± 9.22° vs 10.08 ± 5.42°; *P* < 0.05, *P* < 0.05). During the left-right torsion, around the anteroposterior axis, rotation in group A was higher than that in group B and the control group at L2-3 (9.69 ± 5.94° vs 5.77 ± 4.02°, 4.47 ± 2.00°; *P* < 0.05, *P* < 0.05). In patients with Cobb angle <20°, coupled translation was higher in the degenerated disc group than in the nondegenerated disc group, especially along the anteroposterior axis.

**Conclusion:**

An increase in the coupled rotation of the endplate at the scoliotic apical level in patients with DLS was related to a larger Cobb angle. Moreover, segments with degenerative discs had higher coupled translations in the anteroposterior direction than segments with nondegenerative discs in DLS patients with Cobb angle <20°. These data might provide clues regarding the etiology of DLS and the basis for operative planning.

## 1. Introduction

Degenerative lumbar scoliosis (DLS) was defined as a coronal Cobb angle greater than 10°. DLS is a de novo scoliosis with no previous history and is mainly related to age [1–3], with an incidence of up to 60% [4]. DLS can cause severe symptoms, such as low back pain, radiculopathy, and neurogenic claudication. The pathogenesis of DLS is both complex and controversial. Intervertebral disc degeneration (DD) has also been implicated in the development of DLS [5]. Aebi and Phillips et al. [1, 6] hypothesized that asymmetric loading and degeneration of discs contribute to the development of deformities. Kobayashi et al. [7] reported that asymmetric disc degeneration could predict the incidence of DLS. Murata et al. suggested that DLS could be caused by disc degeneration at any level [8]. In a previous study, asymmetry of the endplates in the midsagittal plane was a risk factor for lumbar disc degeneration [9]. Therefore, the kinematics of the lumbar endplate in DLS patients in vivo should be helpful for the etiology of DLS.

To the best of our knowledge, data on the range of motion (ROM) of the endplate in DLS patients in vivo was scarce. Wang et al. [10] developed a finite element (FE) model to simulate DLS scattering and showed asymmetric loading in the increased asymmetry of the lumbar spine. Zheng et al. [11] also developed an FE model of DLS based on only one patient. There have also been some studies of the human cadaveric spine indicating a relationship between the degenerative disc and ROM of the spine [12–14]. However, they could not reflect the actual status of the lumbar disc and ROM. This study explored the ROM of the lumbar vertebral endplate in vivo to reflect disc deformation using a dual fluoroscopic imaging system. It was reported that the repeatability of the method in reproducing in vivo human spine 6 degree of freedom (DOF) kinematics was <0.3 mm in translation and <0.7° in orientation [15].

This study is aimed at exploring the motion of lumbar endplates in DLS patients with different Cobb angles. Intervertebral DD is believed to have a detrimental effect on the ROM of the spinal segments in degenerative scoliosis [16]. Therefore, we also aimed to investigate the relationship between DD and the ROM of the lumbar vertebral endplates in patients with DLS. We hypothesized that the ROM of the lumbar endplate would be different in DLS patients with different Cobb angles. DD can increase the ROM of the lumbar vertebral endplate in patients with DLS.

## 2. Methods

### 2.1. Subjects and Grouping

In this study, we recruited 42 DLS patients with apical discs at L2-L3 and L3-L4 who were undergoing lumbar surgery, with ages ranging from 41 to 77 years old. We divided the patients into A group with coronal Cobb angle >20° (number:13; 62.00 ± 8.57 years old) and B group with coronal Cobb angle <20° (number:28; 65.79 ± 6.66 years old). We also involved 12 healthy participants reported in the previous study with 52.08 ± 3.18 years old, ranging from 40 to 56 years old, as the control group. L2-L3 and L3-L4 were considered segments around the scoliotic apex, whereas L1-L2, L4-L5, and L5-S1 were considered adjacent apical segments. The institutional review board (IRB) approved this study before initiation. Written consent was obtained prior to any testing. The inclusion criteria were as follows: (1) diagnosed with degenerative adult lumbar scoliosis and the main curve located in the lumbar segments; (2) coronal Cobb angle >10°; and (3) age >40 years. The exclusion criteria were as follows: (1) history of adolescent scoliosis, (2) history of major vertebral trauma, (3) severe joint pain in the lower limbs, (4) leg length discrepancy, (5) history of metabolic disorder, and (6) history of lumbar surgery. In this study, every segment of the lumbar spine (L1-L2, L2-L3, L3-L4, L4-L5, and L5-S1) in all subjects was studied. The magnitude of intervertebral disc degeneration at each segment was determined based on the Pfirrmann classification system [17] (Table 1). Five grades were collected on sagittal T2-weighted images, representing progression from normal disc to severe disc degeneration, in which Pfirrmann grades I and II represented the nondegenerated disc group, whereas Pfirrmann grades III–V represented the degenerated disc group [9]. Disc degeneration was graded by two experienced spine surgeons with more than 5-year experience in degenerative spinal disease. The two surgeons independently and blindly performed the measurements. We selected the mean values of the two surgeons.

### 2.2. Three-Dimensional Models Based on Computed Tomography (CT)

First, we obtained CT images of the lumbar spine of each participant using a CT scanner (Sensation; Siemens, Erlangen, Germany). Images were obtained at a thickness of 0.625 mm. The CT images of the L1-S1 spinal segments were then imported into software (MIMICS 21.0; Materialize, Leuven, Belgium) to build a model of the lumbar spine (Figures 1(a), 1(b), and 1(c)).

### 2.3. Dual Fluoroscopic Imaging System

The position of the lumbar spine was imaged using a dual-fluoroscopic system. Two fluoroscopes (BV Pulsera; Phillips, Bothell, WA, USA) were placed perpendicular to each other. In this way, images of the lumbar spine were simultaneously obtained from two directions. The volunteers were asked to stand between the two perpendicular image intensifiers and make movements, including trunk flexion at 45°, maximal extension, maximal left-right bending, and maximal left-right rotation (Figure 2). A minimum stillness span of 2 s was required for each posture while the two fluoroscopes captured the images. 3D CT-based models of the vertebrae at various body postures were reproduced using the modeling software Rhinoceros (Robert McNeel & Associates, Seattle, WA, USA). Thereafter, the vertebral models were independently translational and rotational in 6DOF until their outlines matched the outlines on the two fluoroscopic images (Figure 2). Using this technique, vertebral endplate positions in vivo were reproduced in different postures.

### 2.4. Coordinate Systems of Vertebral Endplates

Right-hand Cartesian coordinate systems were placed at the center of each vertebral endplate (Figure 1(d)). The center was defined as the volumetric center of the endplate. Based on the geometry of the endplate, the *x*-axis was set parallel to the coronal axis to represent the mediolateral direction and pointed to the left direction. The *y*-axis was set in the horizontal plane and pointed posteriorly to indicate the anteroposterior direction. The *z*-axis was set perpendicular to the transverse plane, representing the cephalad-caudad direction, and pointed in the cranial direction. After moving the vertebrae to different virtual positions, the motion of the inferior endplate of the cranial vertebra was determined relative to that of the superior endplate of the caudal vertebra. Flexion-extension, left-right bending, and left-right torsion of the trunk were compared to the natural upright posture.

### 2.5. Statistical Analysis

A two-way repeated measures ANOVA was used to compare the ROM of the endplates at the L1-L2, L2-L3, L3-L4, L4-L5, and L5-S1 levels. Kinematics was the dependent variable, and vertebral level and activity were the independent variables. The level of statistical significance was set at *P* < 0.05. Another multiway analysis of variance was used to compare the kinematics between patients with different coronal Cobb angles. The participant group was the categorical factor, and the levels and activities were independent variables. When a statistically significant difference was detected, a Newman-Keuls post hoc test was performed, and the level of significance was again set at *P* < 0.05. This was similar in the nondegenerated and degenerated disc groups. Statistical analysis was performed using SPSS version 23 (IBM Corp.) and Prism 7 software (Version 5.01; GraphPad Software Inc., CA, USA).

## 3. Results

### 3.1. Primary Rotations and Translations of Endplates in DLS Patients

During the flexion-extension of the trunk, the mean flexion and extension ranges were 9.42 ± 3.83°, 10.05 ± 5.37°, 11.78 ± 6.46°, 12.59 ± 8.00°, and 12.08 ± 6.73° for the L1-L2, L2-L3, L3-L4, L4-L5, and L5-S1 levels, respectively. During left-right bending of the trunk, the mean left-right bending ranges were 9.44 ± 4.03°, 8.18 ± 4.19°, 9.23 ± 5.39°, 7.97 ± 5.33°, and 8.75 ± 4.95° for the L1-L2, L2-L3, L3-L4, L4-L5, and L5-S1 levels, respectively. During left-right torsion of the trunk, the mean left-to-right twisting ranges were 7.82 ± 4.23°, 7.71 ± 4.73°, 8.86 ± 3.82°, 8.91 ± 6.00°, and 7.92 ± 4.77° for the L1-L2, L2-L3, L3-L4, L4-L5, and L5-S1 levels, respectively. There was no significant difference in the rotational ROM at different levels around the primary axis during the three movements (Figure 3(a)).

### 3.2. Coupled Rotations and Translations of Endplates in DLS Patients

During the flexion-extension of the trunk, along the *z*-axis, translational ROM at L5-S1 was higher than that at L2-L3 and L3-L4 (6.62 ± 3.61 mm vs 4.36 ± 2.55 mm, 5.01 ± 3.19 mm; *P* < 0.05, *P* < 0.05) (Figure 3(d)). Along the *y*-axis, translational ROM at L5-S1 was higher than that at L1-L2 and L2-L3 (8.53 ± 4.76 mm vs 6.04 ± 2.99 mm, 5.45 ± 2.96 mm; *P* < 0.05, *P* < 0.05) (Figure 3(d)). During the left-right bending of the trunk, around the *x*-axis, rotational ROM at L5-S1 was higher than that at L1-L2, L2-L3, L3-L4, and L4-L5 (17.33 ± 9.82° vs 9.68 ± 6.12°, 9.04 ± 5.68°, 8.82 ± 5.28°, 11.41 ± 6.79°; *P* < 0.05, *P* < 0.05, *P* < 0.05, *P* < 0.05) (Figure 3(b)). Along the *y*-axis, translational ROM at L5-S1 was higher than that at L1-L2, L2-L3, and L3-L4 (9.28 ± 6.55 mm vs 4.70 ± 3.07 mm, 6.03 ± 4.35 mm, 5.88 ± 4.31 mm; *P* < 0.05, *P* < 0.05, *P* < 0.05). In addition, along the *z*-axis, translational ROM at L5-S1 was higher than that at L3-L4 (6.65 ± 3.51 mm vs 4.22 ± 2.53 mm; *P* < 0.05) (Figure 3(e)). During left-right torsion of the trunk, around the *x*-axis rotation at L5-S1 was higher than that at L1-L2 (9.12 ± 5.21° vs 7.44 ± 4.26°, *P* < 0.05). Along *x*-axis, translational ROM at L5-S1 was higher than that at L1-L2 and L3-L4 (8.73 ± 4.88 mm vs 5.73 ± 3.75 mm, 5.93 ± 3.22 mm; *P* < 0.05, *P* < 0.05). Along *y*-axis, translational ROM at L5-S1 was higher than other levels (10.73 ± 5.85 mm vs 4.67 ± 2.58 mm, 5.96 ± 4.03 mm, 5.69 ± 3.94 mm, 6.87 ± 3.93 mm; *P* < 0.05, *P* < 0.05, *P* < 0.05, *P* < 0.05). Along *z*-axis, translational ROM at L5-S1 was higher than that at L1-L2, L2-L3, and L3-L4 (6.60 ± 3.98 mm vs 4.06 ± 2.42 mm, 4.59 ± 3.17 mm, 4.27 ± 2.58  mm; *P* < 0.05, *P* < 0.05, *P* < 0.05) (Figure 3(f)).

### 3.3. Comparison of ROMs between Different Cobb Angles and Healthy Subjects (Tables 2 and 3)

During the flexion-extension of the trunk around the *y*-axis, rotation in group A (>20°) was higher than that in the control group at L2-L3 and L3-L4 (10.73 ± 5.11° vs 4.54 ± 2.97°, 8.68 ± 5.21° vs 3.91 ± 2.39°; *P* < 0.05, *P* < 0.05). During the left-right bending of the trunk around the *x*-axis, rotations in groups A and B were higher than those in the control group at L5-S1 (17.52 ± 11.43°, 17.25 ± 9.22° vs 10.08 ± 5.42°; *P* < 0.05, *P* < 0.05). During the left-right torsion of the trunk around the *z*-axis, rotation in the control group was higher than that in groups A and B at L1-L2 (16.48 ± 6.37° vs 8.69 ± 5.56°, 7.43 ± 3.54°; *P* < 0.05, *P* < 0.05) and L5-S1 (17.05°±6.68° vs. 7.69°±5.31°, 8.03°±4.59°; *P* < 0.05, *P* < 0.05). Around the *y*-axis, rotation in group A was higher than that in group B and the control group at L2-L3 (9.69 ± 5.94° vs 5.77 ± 4.02°, 4.47 ± 2.00°; *P* < 0.05, *P* < 0.05).

### 3.4. The Effect of Lumbar Disc Degeneration on ROM of Endplate (Table 4)

During the flexion-extension of the trunk, along the *y*-axis, translation was higher in the degenerated disc group than that in the nondegenerated disc group (6.94 ± 4.09 mm vs 5.37 ± 3.20 mm, *P* < 0.05). In patients with Cobb < 20°, it was significantly different between the degenerated disc group and the nondegenerated disc group along *y*-axis (7.08 ± 4.26 mm vs 5.21 ± 2.91 mm, *P* < 0.05). During left-right bending of the trunk around the *x*-axis, rotation was higher in the degenerated disc group than in the nondegenerated disc group (11.87 ± 7.94° vs 8.82 ± 5.23°, *P* < 0.05). For the patients with Cobb < 20°, along the *y*- and *z*-axis, translations were higher in the degenerated disc group than those in the nondegenerated disc group (6.68 ± 4.88 mm vs 4.68 ± 3.08 mm, 5.36 ± 3.90 mm vs 3.92 ± 2.44 mm; *P* < 0.05, *P* < 0.05). During the left-right torsion of the trunk, along the *x*- and *y*-axis, translations were higher in the degenerated disc group than those in the nondegenerated disc group (*x*: 7.22 ± 4.23 mm vs 5.20 ± 2.67 mm, *y*: 7.28 ± 4.71 mm vs 4.83 ± 3.93 mm; *P* < 0.05, *P* < 0.05). In patients with Cobb < 20°, it is similar along the *x*- and *y*-axis (*x*: 7.19 ± 4.56 mm vs 5.18 ± 2.75 mm, *y*: 7.24 ± 4.60 mm vs 4.59 ± 3.49 mm; *P* < 0.05, *P* < 0.05). However, in patients with Cobb angle >20°, there was no significant difference between the degenerated and the nondegenerated disc groups in the three movements.

## 4. Discussion

The degeneration of the lumbar disc was closely correlated with spinal flexibility in DLS [18]. In this study, we measured the ROM of the vertebral endplates in DLS patients to reflect the biomechanics of the lumbar disc when performing unrestricted weight-bearing activities. The ROM at the lumbosacral junction had a larger ROM of the endplates in coupled rotations and translations than other levels in DLS patients during the three movements. Patients with a Cobb angle >20° had higher coupled rotations at scoliotic apical levels than patients with a Cobb angle <20° and healthy subjects. In DLS patients with Cobb angle <20°, the degenerated disc group had higher coupled translation and rotation than those in the nondegenerated disc group.

In the literature, kinematic measurements of vertebrates in healthy subjects have been investigated in vivo. Shin et al. [19] found that dynamic lumbar axial rotation coupled with lateral binding was segment–dependent. Wu et al. [20] demonstrated that L4–5 and L5–S1 showed larger anteroposterior and proximal–distal translations in healthy participants, respectively. Li et al. [21] found that each vertebral level responded differently to flexion-extension and left-right bending but similarly to left-right twisting in healthy subjects. Some in vivo studies have reported the kinematics of the lumbar spine in patients with low back pain [22], degenerative disc disease [23], and degenerative spondylolisthesis [24]. There have also been some studies of the human cadaveric spine indicating a relationship between the degenerative disc and ROM of the spine [12–14]. Fujiwara et al. [13] noted that segmental motion initially increases with degeneration, similar to our study. However, kinematics of the lumbar spine in DLS patients has only been conducted using the FE model. Wang et al. [10] built FE models with three different Cobb angles modified from a normal lumbar spine and found that asymmetric loading on facet joint contact forces accelerates asymmetry in the lumbar spine. However, in vivo studies on DLS kinematics were scarce.

In our study, the difference in vertebral endplate ROM between patients with DLS and healthy participants was mainly in rotational ROM. In patients with DLS, the ROM of the endplates around the apical disc was larger in coupled motions. At the adjacent levels, particularly in the lumbosacral joint, the ROMs of the coupled motion were high. Moreover, patients with a larger coronal Cobb angle had larger coupled motions at the scoliotic apical level, which might induce more changes in adjacent biomechanics after fusion to the scoliotic apical level. Rustenburg et al. [16] also found a positive correlation between the Cobb angle and coupled motions, suggesting that the magnitude of coupled motions increased as the disease progressed in the cadaveric spines. This implied that the coupled motions increased as the asymmetry of the spine increased at all levels, which might be due to less alignment in the local axes [25]. In addition, Rustenburg et al. [16] reported that spines with DLS tend to be stiffer and less flexible. This might be related to the larger coupled motion around the apical level. In Schlösser et al.'s study [26], the degree of torsion also correlated significantly with the Cobb angle, and they thought that morphological modifications of vertebrates were rather a consequence of the deformity. In addition, the anatomical deformation trend of vertebral endplates in Schlösser et al.'s article [26] might be caused by the increased coupled motion of DLS. Generally, a greater increase in coupled motion in patients was related to a larger Cobb angle. These data may help explore the etiology of DLS.

Kobayashi et al. [7] found that asymmetric disc degeneration could be a predictive factor for the incidence of DLS using logistic regression analysis in a community-based cohort. Primary degeneration of the disc is considered an initiating event of secondary deterioration of the facets and ligaments [27]. In our study, degenerative discs had higher coupled motions than nondegenerative discs in patients with DLS, particularly in patients with a small Cobb angle. This might be related to the degenerative disc located around the coronal scoliotic apex. However, increased coupled motion might also increase disc degeneration. Murata et al. [8] studied human cadaveric spinal motion segments and suggested that all lumbar interval spaces from L1–L2 to L5–S1 could trigger degenerative lumbar scoliosis. In our study, we found that the coupled motion of the degenerative disc at any level was larger, which might be related to Murata et al.'s results. Ellingson et al. [12] found positive correlations between Pfirrmann grade and axial rotation ROM. Schmidt et al. [14] reported increased ROM for axial rotation, flexion-extension, and lateral bending with increased disc degeneration. Fujiwara et al. [13] found that degeneration increased the ROMs in all rotational modes in discs with moderate degeneration, similar to our study. Murata et al. [8] suggested that disc degeneration might cause wedging progression. When the angle of the consequential wedging, which was bent to the side opposite the initial wedging to preserve balance, became larger than that of the initial wedging, the lumbar spine might attempt to maintain balance by making the initial wedging progress [8]. The increased coupled motion of the degenerative disc might be associated with sequential wedging to maintain balance. In Bao et al.'s study [28], the regional lumbar disc Pfirrmann score was also strongly correlated with the Cobb angle on the coronal plane. In our study, we found that degenerative discs in DLS patients with a coronal Cobb angle of <20° had larger coupled motions. A possible reason might be that patients with mild DLS had a more flexible ability to compensate for balance than patients with severe DLS, which also contributed to the development of DLS. Therefore, it should be considered cautiously about the fixed levels when there is already severe disc degeneration at the adjacent segment, even in DLS patients with a small Cobb angle, to avoid future failure at adjacent levels.

Our study had some limitations. First, the sample size of the patients with severe DLS was relatively small. Furthermore, the patients involved in the study were specifically selected with apical discs at the L2-L3 and L3-L4 levels, which represented only a portion of all patients with DLS. Finally, although we attempted to make the same movements for everyone, DLS patients might move more or less differently because of back pain.

## 5. Conclusions

In general, this study used an in vivo technique to quantify the abnormal motion of the vertebral endplates in DLS patients during various postures. An increase in the coupled motion of the endplate in DLS patients at the scoliotic apical level was related to a larger Cobb angle. Moreover, the segment with degenerative disc had higher coupled translations in the anteroposterior direction than the nondegenerative disc in DLS patients with Cobb angle <20°. These data might provide clues regarding the etiology of DLS and the basis for operative planning.

## Figures and Tables

**Figure 1:** (a) Digitized contours of lumbar vertebrae in coronal plane. (b, c) Three-dimensional anatomic vertebral model constructed from the computed tomography. (d) Anatomic coordinate system to measure kinematics of the endplates.

**Figure 2:** Each 3D vertebral model was separately translated and rotated until their contours matched the corresponding vertebral bony outline captured on the 2 fluoroscopic images.

**Figure 3:** Range of motion of endplates in DLS patients during standing up and along three principal axes under (a, d) flexion-extension, (b, e) bending, and (c, f) torsion of the trunk. The symbols (^∗^, +, △) represent statistical significance on comparison of different level (*P* < 0.05).

**Table 1:** Pfirrmann classification of disc degeneration in DLS Patients (Cobb > 20° and Cobb < 20°).

	L1-L2	L2-L3	L3-L4	L4-L5	L5-S1
A group	2.92 ± 0.86	3.08 ± 0.64	3.38 ± 0.96	3.69 ± 0.63	3.69 ± 0.95
Range of grade	1-5	2-4	2-5	3-5	2-5
B group	2.72 ± 0.96	2.79 ± 0.68	3.31 ± 0.81	3.66 ± 0.86	3.66 ± 0.94
Range of grade	2-4	2-4	2-5	3-5	2-5

The values were presented as mean ± SD. DLS: degenerative lumbar scoliosis; A group: coronal Cobb > 20°; B group: coronal Cobb < 20°.

**Table 2:** Comparison of rotation ranges (°) between normal participants and DLS patients (Cobb > 20° and Cobb < 20°).

Level	L1-L2			L2-L3			L3-L4			L4-L5			L5-S1		
Axis	*x*	*y*	*z*	*x*	*y*	*z*	*x*	*y*	*z*	*x*	*y*	*z*	*x*	*y*	*z*
Flexion-extension															
A group	10.09 ± 4.56	8.82 ± 4.88	3.75 ± 3.92	9.26 ± 4.43	10.73 ± 5.11	4.64 ± .3.92	11.20 ± 5.94	8.68 ± 5.21	4.14 ± 2.73	13.75 ± 8.48	6.90 ± 3.77	4.63 ± 4.56	12.21 ± 7.20	9.07 ± 5.55	3.56 ± 4.81
B group	9.12 ± 3.51	7.01 ± 4.22	3.06 ± 2.12	10.40 ± 5.78	7.24 ± 4.13	3.20 ± 4.59	12.04 ± 6.76	6.42 ± 4.52	3.52 ± 3.15	12.07 ± 7.89	7.53 ± 7.55	3.06 ± 2.95	12.02 ± 6.63	6.78 ± 3.72	3.52 ± 2.44
Normal	9.40 ± 3.84	7.05 ± 4.22	3.43 ± 2.73	9.40 ± 5.08	7.48 ± 4.62	3.52 ± 4.15	11.37 ± 5.94	6.41 ± 4.56	3.73 ± 3.01	11.83 ± 7.46	7.06 ± 6.02	3.56 ± 3.91	12.46 ± 6.32	7.01 ± 4.16	4.58 ± 3.96
Left-right bending															
A group	12.72 ± 7.92	9.01 ± 3.75	5.77 ± 4.57	9.51 ± 5.96	10.52 ± 4.94	6.20 ± 5.57	9.32 ± 4.84	8.51 ± 5.43	3.91 ± 2.93	11.75 ± 7.13	6.19 ± 4.38	4.23 ± 2.86	17.52 ± 11.43	8.65 ± 4.87	6.99 ± 6.78
B group	8.32 ± 4.67	9.63 ± 4.19	5.39 ± 4.84	8.82 ± 5.65	7.13 ± 3.40	2.99 ± 3.34	8.59 ± 5.53	9.55 ± 5.43	5.05 ± 4.82	11.25 ± 6.75	8.77 ± 5.59	3.79 ± 2.78	17.25 ± 9.22	8.79 ± 5.07	3.81 ± 2.37
Normal	7.53 ± 3.76	9.11 ± 4.28	4.60 ± 4.70	8.25 ± 4.36	5.96 ± 2.54	4.05 ± 3.23	9.78 ± 5.07	8.50 ± 4.14	4.68 ± 4.93	8.34 ± 4.50	5.24 ± 3.44	3.47 ± 2.79	10.08 ± 5.42	10.06 ± 4.31	7.85 ± 4.38
Left-right torsion															
A group	9.55 ± 3.04	9.39 ± 5.94	8.69 ± 5.56	10.53 ± 6.24	9.69 ± 5.67	9.95 ± 6.74	6.21 ± 4.44	8.22 ± 5.63	10.48 ± 4.10	8.36 ± 4.74	7.33 ± 2.19	11.17 ± 7.91	10.66 ± 7.66	6.01 ± 5.93	7.69 ± 5.31
B group	6.49 ± 4.42	6.76 ± 4.33	6.71 ± 3.15	8.72 ± 5.89	5.77 ± 4.02	6.71 ± 3.15	9.79 ± 5.93	7.25 ± 4.43	8.13 ± 3.52	9.47 ± 5.45	7.37 ± 4.80	7.89 ± 4.74	11.45 ± 8.03	7.87 ± 4.73	8.03 ± 4.59
Normal	8.74 ± 7.66	5.71 ± 3.30	16.48 ± 6.37	7.62 ± 3.89	4.47 ± 2.00	11.29 ± 4.91	10.74 ± 5.10	5.93 ± 3.87	15.64 ± 6.29	8.18 ± 7.34	4.76 ± 2.93	11.79 ± 7.27	10.18 ± 5.27	5.49 ± 3.67	17.05 ± 6.68

Mean values were presented as ± standard deviation. Rotation around axis: *x*, *y*, and *z*. DLS: degenerative lumbar scoliosis; *x*: mediolateral.axis; *y*: anteroposterior axis; *z*: craniocaudal axis; A group: coronal Cobb > 20°; B group: coronal Cobb < 20°.

**Table 3:** Comparison of translation ranges (mm) between normal participants and DLS patients (Cobb > 20° and Cobb < 20°).

Level	L1-L2			L2-L3			L3-L4			L4-L5			L5-S1		
Axis	*x*	*y*	*z*	*x*	*y*	*z*	*x*	*y*	*z*	*x*	*y*	*z*	*x*	*y*	*z*
Flexion-extension															
A group	5.37 ± 3.71	5.75 ± 3.68	5.47 ± 2.74	7.31 ± 3.78	5.18 ± 2.34	5.31 ± 2.96	5.14 ± 2.81	6.29 ± 3.39	5.63 ± 3.47	5.57 ± 3.13	6.03 ± 3.47	4.52 ± 3.02	6.66 ± 2.84	9.47 ± 4.61	6.78 ± 2.99
B group	6.15 ± 4.33	6.17 ± 2.69	5.25 ± 3.77	5.83 ± 4.59	5.57 ± 3.23	3.93 ± 2.27	5.01 ± 3.72	7.24 ± 5.02	4.25 ± 2.29	4.96 ± 3.47	6.25 ± 3.79	5.22 ± 3.29	7.58 ± 4.98	8.11 ± 4.84	6.54 ± 3.89
Normal	3.97 ± 1.69	4.58 ± 3.16	4.05 ± 1.90	4.28 ± 2.03	4.76 ± 3.31	3.58 ± 2.44	4.61 ± 2.78	6.12 ± 4.45	4.59 ± 2.40	4.26 ± 1.39	6.15 ± 4.75	5.63 ± 2.69	5.99 ± 4.77	9.68 ± 7.18	5.58 ± 2.55
Left-right bending															
A group	5.22 ± 4.15	4.28 ± 2.40	3.53 ± 1.91	6.01 ± 3.76	6.95 ± 5.32	5.85 ± 3.84	5.87 ± 3.64	7.22 ± 5.86	3.90 ± 2.06	6.45 ± 4.38	6.61 ± 3.68	4.84 ± 2.53	7.28 ± 4.20	9.94 ± 6.05	6.90 ± 4.18
B group	5.47 ± 2.63	4.89 ± 3.35	4.98 ± 5.57	5.46 ± 4.19	5.61 ± 3.87	4.14 ± 3.22	5.29 ± 3.30	5.28 ± 3.35	4.36 ± 2.73	4.53 ± 3.46	6.43 ± 3.74	5.19 ± 2.48	5.98 ± 3.97	8.98 ± 6.84	6.53 ± 3.25
Normal	5.35 ± 2.95	5.22 ± 2.51	4.71 ± 2.22	5.77 ± 3.25	7.58 ± 2.82	3.53 ± 2.12	5.59 ± 2.04	4.79 ± 2.87	5.04 ± 2.41	4.93 ± 2.15	7.55 ± 4.83	6.20 ± 4.79	8.76 ± 6.56	7.19 ± 5.94	4.93 ± 3.08
Left-right torsion															
A group	5.28 ± 2.13	5.38 ± 2.79	4.35 ± 2.30	7.98 ± 5.05	5.18 ± 4.24	5.46 ± 4.45	5.60 ± 2.78	5.42 ± 4.55	3.82 ± 1.96	7.02 ± 3.71	6.43 ± 3.12	5.49 ± 4.51	8.96 ± 4.84	12.98 ± 5.40	6.50 ± 3.30
B group	5.93 ± 4.31	4.36 ± 2.47	3.93 ± 2.49	5.84 ± 3.49	6.31 ± 3.96	4.20 ± 2.39	6.08 ± 3.43	5.81 ± 3.71	4.48 ± 2.82	7.27 ± 4.70	7.07 ± 4.28	4.81 ± 2.99	8.61 ± 4.98	9.73 ± 5.86	6.65 ± 4.30
Normal	6.37 ± 3.32	4.78 ± 3.21	5.12 ± 4.01	4.64 ± 3.54	5.85 ± 2.69	5.11 ± 2.57	6.37 ± 3.47	4.68 ± 2.72	2.96 ± 2.17	5.26 ± 2.63	6.52 ± 4.05	5.42 ± 4.17	7.68 ± 4.96	9.25 ± 6.79	3.45 ± 2.40

Mean values were presented as ± standard deviation. Rotation around axis: *x*, *y*, and *z*. DLS: degenerative lumbar scoliosis; *x*: mediolateral axis; *y*: anteroposterior axis; *z*: craniocaudal axis; A group: coronal Cobb > 20°; B group: coronal Cobb < 20°.

**Table 4:** Comparison of translation ranges between normal participants and DLS patients (Cobb > 20° and Cobb < 20°).

Number		A group		*P* value	B group		*P* value
		Nondegenerative disc	Degenerative disc		Nondegenerative disc	Degenerative disc	
		10	55		32	113	
Rotations (°)							
Flexion-extension	*x*	10.93 ± 4.68	11.37 ± 6.61	0.840	9.60 ± 4.88	11.56 ± 6.61	0.121
	*y*	8.24 ± 4.67	8.95 ± 5.02	0.676	6.82 ± 3.94	7.05 ± 5.24	0.813
	*z*	4.48 ± 3.17	4.08 ± 4.09	0.737	3.16 ± 3.77	3.31 ± 2.94	0.831
Left-right bending	*x*	9.31 ± 5.21	12.68 ± 8.47	0.192	8.66 ± 5.31	11.47 ± 7.67	0.063
	*y*	9.25 ± 5.10	8.45 ± 4.75	0.629	7.69 ± 3.69	9.08 ± 5.07	0.149
	*z*	6.39 ± 4.02	5.25 ± 4.92	0.421	4.48 ± 3.97	4.13 ± 3.80	0.672
Left-right torsion	*x*	8.15 ± 3.17	9.23 ± 5.88	0.602	8.70 ± 5.55	9.32 ± 6.38	0.608
	*y*	10.03 ± 8.05	7.78 ± 4.64	0.168	6.64 ± 3.67	7.10 ± 4.68	0.625
	*z*	8.90 ± 5.34	9.72 ± 6.16	0.610	7.17 ± 3.02	7.77 ± 4.17	0.528
Translations (mm)							
Flexion-extension	*x*	5.85 ± 3.95	6.04 ± 3.20	0.893	5.56 ± 4.66	6.01 ± 4.21	0.579
	*y*	5.89 ± 4.15	6.66 ± 3.74	0.569	5.21 ± 2.91	7.08 ± 4.26	0.019^∗^
	*z*	4.88 ± 3.02	5.67 ± 3.06	0.476	5.17 ± 3.56	5.00 ± 3.20	0.797
Left-right bending	*x*	4.16 ± 4.90	6.53 ± 3.71	0.061	4.80 ± 2.88	5.50 ± 3.70	0.338
	*y*	5.66 ± 4.12	7.25 ± 5.20	0.327	4.68 ± 3.08	6.68 ± 4.88	0.035^∗^
	*z*	3.75 ± 3.10	5.23 ± 3.20	0.220	3.92 ± 2.44	5.36 ± 3.90	0.041^∗^
Left-right torsion	*x*	5.30 ± 2.52	7.27 ± 4.16	0.168	5.18 ± 2.75	7.19 ± 4.56	0.016^∗^
	*y*	5.61 ± 5.24	7.35 ± 4.96	0.272	4.59 ± 3.49	7.24 ± 4.60	0.004^∗^
	*z*	4.90 ± 2.27	5.17 ± 3.68	0.813	4.19 ± 2.51	4.99 ± 3.34	0.228

Mean values were presented as ± standard deviation. Rotation around axis: *x*, *y*, and *z*. ^∗^, *P* value < 0.05. DLS: degenerative lumbar scoliosis; *x*: mediolateral.axis; *y*: anteroposterior axis; *z*: craniocaudal axis; A group: coronal Cobb > 20°; B group: coronal Cobb < 20°.

## Data Availability

The datasets used and/or analysed during the current study were available from the corresponding author on reasonable request.
